RETRACTED

# Packaging Design Based on Deep Learning and Image Enhancement

**DOI:** 10.1155/2022/9125234

**Published:** 2022-08-01

**Authors:** Jinping Liu

**Affiliations:** Jilin University of Architecture and Technology, Changchun 130111, China

## Abstract

Packaging design is an important part of product design. How to improve the efficiency of packaging design is a problem that must be considered in product design. Existing packaging design methods require a lot of human and material resources. In view of this situation, this paper proposes a packaging design method based on deep learning. This paper innovatively proposes a packaging design model based on deep convolution generative adversarial networks (DCGAN). This paper constructs a dataset of packaging design schemes and trains the proposed DCGAN model. The results show that the packaging design generated by the model proposed in this paper can get a score similar to that of the expert design scheme, which proves the effectiveness and rationality of the proposed model. In addition, in order to further improve the imaging quality of packaging design images, this paper proposes a packaging design image enhancement method based on visual communication technology. The packaging design image enhancement processing is carried out through the guided filtering method, and the visual communication optimization and edge pixel fusion methods are used to decompose the multidimensional scale features of the packaging design image under the visual communication technology to realize the packaging design image enhancement processing. The simulation results show that the method used for packaging design image enhancement processing has better visual communication ability, higher degree of image information fusion, and improved packaging design effect.

## 1. Introduction

Appearance design is one of the key points of product design for packaging. When designing packaging, factors such as packaging materials and structure, the cultural connotation of the brand, the use of colors, and the fit of the festival theme need to be considered [1]. This complicates the design of the appearance of packaging products, increases the design difficulty, and increases time and labor costs [2].

With the development of packaging design technology, combined with computer vision image analysis methods to optimize packaging design and improve the ability of packaging design image fusion analysis, the research on related packaging design image processing methods has received great attention. The packaging design image is analyzed by the computer three-dimensional visual feature analysis method, the edge contour feature quantity of the packaging design image is extracted, and the packaging design image is processed by the method of texture distribution and information enhancement [3]. This new design method based on computer vision helps to improve the effect of packaging design, and the related research on image enhancement methods for packaging design has received great attention. One of the main tools of current image processing is the backpropagation neural network, which is the core model of deep learning [4].

RETRACTED

The image enhancement processing of packaging design under visual communication technology is based on the sampling and information fusion of packaging design images, and the information fusion and feature extraction model of packaging design images are constructed [5]. Through image visual information enhancement processing, the envelope feature detection of packaging design images is carried out, and the distribution set of packaging design visual communication features is analyzed [6]. Through the reconstruction of 3D information under computer vision and the use of optical information sensing technology, the image processing of packaging design is realized [7]. The packaging design image enhancement method based on Harris corner detection and the packaging design image enhancement method based on Harris corner detection are used to construct a three-dimensional distribution model of packaging design image information, but the visual communication performance of traditional methods for packaging design is not high [8].

The appearance design of image-driven packaging products can be regarded as an image-to-image style transfer problem, but there are few reports on the combination of deep learning and packaging design [9]. Deep learning can generate renderings of appearance designs based on input sketches, which not only provides inspiration for color matching and texture selection for the appearance design work of packaging products but also provides a reference for subsequent personalized modification work [9]. In order to effectively apply image processing techniques to packaging design, appropriate models need to be selected. In 2014, Steenis et al. and others proposed the generative adversarial network (GAN) and applied it to image translation tasks. The research results show that GAN has achieved better results than the traditional convolutional neural networks (CNN). Most GANs are based on paired or unpaired input images, learn and generate output images corresponding to the target image, so that the generated image has the texture of the input image and the content of the target image [6].

Therefore, this paper proposes a GAN-based packaging product design method in order to provide a new model for packaging design.

RETRACTED

## 2. Model and Method

### 2.1. Generative Adversarial Networks

A generative adversarial network (GAN) is a deep learning model that can achieve good results on unsupervised learning. GAN is a new framework for estimating and generating models in the adversarial process, and its main components are divided into two parts: a generative model (G) and a discriminative model (D).

The generative model G generates new samples that are as close to the real samples as possible by analyzing the underlying data distribution of the real data samples. The discriminant model D judges whether a sample comes from the training data by outputting a probability value. When the probability value is greater than 0.5, it is true, and otherwise, it is false. The model framework finds a balance point through continuous training, so that both can be improved. At this time, the discriminator D cannot distinguish whether the data come from real data. The model structure of the adversarial neural network is shown in Figure 1.

As shown in Figure 1, the network on the right is the discriminant network D. Its structure is similar to the traditional cyclic convolutional network. The probability value of the output is obtained through the input data set *X* to determine whether the input comes from the real data set. If the output probability value is >0.5, it means that the input comes from the real data set; if the output probability value is <0.5, it means that the input is newly generated data. The advantage of the discriminative network is that it can help us understand the distribution of image data, but it also has the disadvantages of very high acquisition cost, large amount of data, and consumption.

The generative network G is the network on the left in Figure 1, its input is a set of random noise *Z*, and the output is new data *G*(*z*) that is as close as possible to the real data distribution. Its network structure can be regarded as the inverse structure of the discriminant network, and through several layers of deconvolution calculations, new data are generated directional or nondirectional. Whether the generative network can obtain high-quality results depends on how to optimize the structure and parameters of the generative network. Training and sampling data in a generative network can measure how well a researcher can analyze and compute high-dimensional probability distributions.

### 2.2. Basic Structure of DCGAN

The deep convolutional generative adversarial network (DCGAN) introduced the convolutional network into the structure of GAN for the first time and used the powerful feature extraction ability of the convolutional layer to improve the learning effect of GAN. DCGAN has proved to be robust and stable in practice. The input layer consists of a 100-dimensional Gaussian noise *z* and a one-hot encoded product image *y*, followed by a matrix variable dimension layer and 4 convolutional layers. After the input layer passes through the matrix variable dimension layer, the output dimension size is 4 × 4 × 1024, and then, it is input into the following 4 fractional stride convolutional layers, where the convolution kernel size is 5 × 5 and the stride is 2. 4 fractional stride convolutional layers conv1, conv2, conv3, and conv4 increase the length and width of the output dimension, while decreasing the depth, respectively, 8 × 8 × 512, 16 × 16 × 256, 32 × 32 × 128, 64 × 64 × 3, the final output from the fractional stride convolutional layer conv4 is the design of the generated packaging. The input layer in the discriminant model consists of 3 parts: the one-hot encoded product image, the real data product image, and the generative design sample image output by the generative model. Then, there are 4 convolutional layers conv1, conv2, conv3, and conv4 to reduce the dimension length and width of the output, while increasing the depth, respectively, 32 × 32 × 64, 16 × 16 × 128, 8 × 8 × 256, 4 × 4 × 512, and finally, output the probability value through a fully connected layer of the sigmoid function to determine whether the image is a real sample that satisfies the packaging.

RETRACTED

The details of the DCGAN experiment should pay attention to the following steps:

  Step 1: the preprocessing performed in the experiment is simply to scale the training image to the range [−1, 1] of the tanh activation function
  Step 2: mini-batch training, the batch size is 16
  Step 3: all weight values are initialized from a normal distribution centered at 0 with a standard deviation of 0.02
  Step 4: in LeakyReLU, the slope of all models is set to 0.2
  Step 5: DCGAN uses Adam optimizer to speed up training
  Step 6: the learning rate of the Adam optimizer is set to 0.0002
  Step 7: reduce the momentum parameter *β*1 from 0.9 to 0.5 to prevent oscillation and instability

### 2.3. Packaging Image Dataset

In order to reduce cost consumption and generate results quickly, this research will build a small packaging image dataset containing about 2,000 icons, and the data sources are Google Images and Baidu Images. Python's scratch tool is used to obtain packaged images.  Figure 2 shows a thumbnail of some packaging design images of the self-created dataset.

In order to expand the number of datasets and meet the needs of deep learning model convergence, this paper adopts the following data augmentation methods:

1. Translation: move all the pixels in the image along the horizontal or vertical direction, or both directions. It should be noted that the image will vacate a part of the area after translation, and the filling method should be selected according to the actual situation of the data.
2. Cropping: randomly select a part of the image to crop, usually enlarge this part to the original size.
3. Rotation: rotate the image clockwise or counterclockwise. When rotating at any angle (not 180 degrees), fill the empty position.
4. Flip: flip the image horizontally or vertically.
5. Zoom: enlarge or reduce the image by a certain ratio. After the image is enlarged, it usually needs to be cut to the original size. After the image is reduced, select an appropriate method to fill it.
6. Add noise: randomly add noise to the picture, common ones are Gaussian noise.
7. Color transformation: increase or decrease the components of certain colors on the picture.

RETRACTED

In addition, this paper also uses the SamplePairing data to enhance the crime. SamplePairing is to randomly synthesize a new sample in the form of averaging the pixels of the two images in the training set after conventional data enhancement (flip, crop, rotation, etc.), and the label is one of the labels of the original image.

### 2.4. Model Implementation Steps

The implementation steps of the model are as follows:

1. Set basic parameters, including the storage path of the packaging image dataset, the generation path of the new packaging image, the learning rate of the training network, and the number of samples processed in each loop.
2. Packaging image preprocessing and data structure transformation: where the data transformation is to convert a two-dimensional icon into an array of tensors suitable for matrix calculations.
3. By means of data set classification or computer-aided recognition, conditional labels are introduced to adjust the iterative direction of the network model and the effect of packaging image generation.
4. The algorithm using the self-attention mechanism identifies the packaged image data, obtains high-level icon features, combines with the original input, and passes it to the generation network and the discriminant network.
5. Build generation network and discrimination network: the generation network is a multilayer deconvolution function, and the received noise and condition labels are input to generate new icons. The discrimination network is a multilayer convolution function, the received sample icon, generated icon, and condition label are input, and the probability value is output.
6. Define loss function: the loss function of the generated network is only related to the generated packaging image and its probability. The loss function of the discriminant network needs to average the probability values of the sample image, the generated image, and each source.
7. Expand the loop, and use the backpropagation algorithm to update the network weight value at the end of each loop.
8. Record the network model regularly and output the packaging image.

RETRACTED

The basic framework and implementation flow of the packaging design generation countermeasure network are shown in Figure 3.

## 3. Image Enhancement and Optimization Method for Packaging Design

### 3.1. Feature Analysis and Automatic Aggregation Matching

A low-pass filter detection method is used for feature analysis and automatic aggregation matching of visual communication of packaging design. Through the guided filtering method, the packaging design image is enhanced, and the adaptive matching function of the packaging design image is

(1) $$\begin{array}{c} \text{fitness}\left(z\right)=\left\{\begin{array}{cc} 1+Ef\left(z\right), & \text{if feasible},\\ f\left(z\right), & \text{otherwise}. \end{array}\right. \end{array}$$

In the formula, *f*(*z*) is the packaging design image enhancement processing function; *E* is the packaging design image aggregation function.

In the pixel cluster of the packaging design image, the statistical feature distribution set of the packaging design image is obtained as

(2) $$\begin{array}{c} K=\frac{e^{\ln\;a}}{\sqrt{a}}+u\left(f\left(z\right)+bW\right). \end{array}$$

In the formula, *u*(·) is the pixel difference fusion model of the packaging design image.

In the multiscale packaging design image distribution set, the cost function of the packaging design image feature category focus is obtained. Through rough set feature matching, the frequency factor of the packaging design image is obtained as

(3) $$\begin{array}{c} U=\frac{\tau C_{\max}C_{\min}/K}{C_{0}\tau }. \end{array}$$

Among them, *C*_0_ is the fitness coefficient of the packaging design image; *C*_min_ and *C*_max_ are the lowest and highest cost functions of the packaging design image, respectively; *τ* is the matching time.

Through multiscale decomposition, the block fusion model of the packaging design image is obtained as

(4) $$\begin{array}{c} L=W⊗U+a. \end{array}$$

In the formula, ⊗ is the fuzzy convolution operator of the packaging design image; *U* is the focusing function of the packaging design image; *a* is the fusion factor.

According to the above analysis, a block detection model of the packaging design image is constructed, and the focused fusion output of the packaging design image is obtained as

(5) $$\begin{array}{c} M=\sum_{i=-\infty }^{0}\int_{j=0}^{+\infty }L\left(\tau -i\gamma +j\gamma \right)\text{d}\gamma . \end{array}$$

In the formula, *γ* is the time sampling interval for the aggregation and matching of packaging design image features.

RETRACTED

According to the above analysis, an optimized feature matching model for packaging design images is established to improve the image enhancement ability.

### 3.2. Packaging Design Image Enhancement

Based on the above-mentioned optimized feature matching model, using visual communication optimization and edge pixel fusion methods, an enhanced three-dimensional reconstruction model of packaging design images is established, and the feature quantities of semantic information in the gray area of packaging design images are obtained as follows:

(6) $$\begin{array}{c} \text{pixel}\_\chi =\max\left(u\sum \left(L-k\right)\right). \end{array}$$

In the formula: *u* is the edge pixel of the packaging design image; *L* is the gray area function of the packaging design image; *k* is the reconstructed feature quantity of the packaging design image.

A low-resolution and high-resolution information fusion model of packaging design image enhancement is established, and the gray features of packaging design image enhancement are decomposed through the spatial region fusion method, and the fuzzy correlation degree of the packaging design image is obtained as *ϕ*, with (*x*, *y*) as the center, and the packaging design is carried out. The edge scale decomposition of the image is expressed as follows:

(7) $$\begin{array}{c} \text{pixel}\_\kappa =\max\left(a\sum \left(\phi L-k\right)\right). \end{array}$$

If pixel_*χ* < pixel_*κ*, the optimal matching and information transmission of the packaging design image are controlled, and the template matching function for the visual communication of the packaging design is obtained as

(8) $$\begin{array}{c} \omega =\frac{\mu /\pi -\lambda_{2}}{\lambda_{1}}. \end{array}$$

In the formula, *μ* is the information enhancement feature quantity of the visual communication of the packaging design; *λ*_1_ and *λ*_2_ are the long and short edge packaging scales, respectively.

Through the edge feature decomposition of the packaging design image, the information enhancement output is obtained as follows:

(9) $$\begin{array}{c} N=\sum_{i=1}\omega \left(\varepsilon_{i}C_{i}\right)-h\left(V_{i}\right). \end{array}$$

In the formula: *h*(*V*_*i*_) is the edge feature decomposition function; *ω*(*ε*_*i*_*C*_*i*_) is the information enhancement coefficient.

Using adaptive feature detection decomposition and visual communication technology, the filtering enhancement function of the packaging design image is obtained as follows:

(10) $$\begin{array}{c} D=N+\sum_{\sigma =1}^{m}\frac{\hat{x}\left(n\right)}{u_{\sigma }\left(n\right)}. \end{array}$$

In the formula, *A* is the edge focus function of the packaging design image; *B* is the feature decomposition scale of the packaging design visual communication; *C* is the pixel intensity; and *D* is the energy coefficient of the packaging design visual communication.

RETRACTED

In the formula, $\hat{x}\left(n\right)$ is the edge focus function of the packaging design image; *m* is the feature decomposition scale of the packaging design visual communication; *u*_*σ*_(*n*) is the pixel intensity; and *σ* is the energy coefficient of the packaging design visual communication.

Through the method of neighborhood interpolation compensation, the visual compensation function of packaging design is obtained as follows:

(11) $$\begin{array}{c} F=\overset{n}{\underset{w=1}{\sum }}\frac{Dw}{\sum_{i=-\infty }^{0}\int_{j=0}^{+\infty }L\left(\tau -i\gamma +j\gamma \right)\text{d}\gamma }. \end{array}$$

In the formula, *w* is the information enhancement coefficient of packaging design.

## 4. Experiments and Results

### 4.1. Running Environment

This research and design practice is mainly realized with the help of the Python programming language. Python is a mainstream deep learning language with simple logic and is suitable for data operation and analysis. This time, the Macintosh OS Mojave operating system is used, together with the installation of the Python 3 5 complete function library.

The library functions mainly used in this research include the following:

1. TensorFlow: an open-source framework for deep learning. Its working principle is to convert files of various formats into N-dimensional array matrices and write the network model structure in a form similar to drawing a flowchart. Depending on the purpose of the user, the working mode of the CPU or GPU can be selected. Since its release, Tensorflow has been downloaded and used by enterprises and individual developers.
2. Pillow (PIL): integrated image processing function library that supports a variety of image formats and sizes. With the help of the Pillow function, basic operations such as image reading, image editing, and image storage can be implemented.
3. NumPy: represents the combination of Number and Python. It is mainly used for matrix operations on tensor arrays and has a fast response effect for processing large matrices.
4. SciPy: indicates the combination of scientific science and Python, often used together with NumPy. It is a function library that extends the definition of NumPy and is mainly responsible for processing NumPy arrays under matrix calculations.
5. OpenCV: a computer vision function library that supports multiple programming languages and operating systems and has the advantages of convenient use, accurate operation, and fast efficiency. Researchers can use OpenCV for image recognition, image processing, and video editing.
6. Matplotlib is used to implement the drawing and display of icon images and geometric figures. It has the advantages of small memory occupation and fast generation speed.

RETRACTED

### 4.2. Simulation Training and Results of the Model

Suppose there are several original line segments real_lines distributed in the space, some are high and some are low, but the curvatures formed are the same. The generative adversarial network can learn the curvature changes of these line segments and generate new curves “new_lines” that are similar to the curvature of the original line segments through training.

#### 4.2.1. Setting Parameters

The first is the most important parameter “Batch_Size” in deep learning, which indicates the number of samples used in each training and determines the convergence direction of the entire network model.

If the batch size is set to the total amount of data contained in the dataset, it is called a “full dataset.” At each training, the network processes every piece of information in the sample dataset, which ensures that the input distribution fits the overall picture. However, the scale and number of datasets are relatively large, and loading all the data at one time will increase the training cost and even cause memory overflow problems. If the batch size is set to 1, only one sample of data is trained in each loop. At this time, each new cycle will cause the convergence direction to proceed in the gradient direction of the respective samples, which affects the normal iteration of the network.

Therefore, in formal training, it is recommended to choose medium size batch values, such as 32, 64, and 128. Training with these data computes gradients that are almost the same as those trained on all data and avoids out-of-memory issues. In this simulation, the batch size is set to 64, the number of cycles Epoch is set to 5000, the number of points connected to each line segment is set to 30 (to ensure the smoothness of the line segment), and the generation interval of the original line segment is [1, 2].

#### 4.2.2. Define the Training Network

In the definition of the loss function of the generative network and the discriminant network, the learning rate (Learning Rate) is introduced as the speed of the function change. In general, the larger the learning rate, the faster the training; however, a fast training speed does not mean that the training model is successful, and too fast a speed may lead to abnormal convergence of the function.

RETRACTED

The generated training network is defined as

(12) $$\begin{array}{c} \text{Train}\_G=\text{optimizer}\left(\text{LR}\right).\text{minimize}\left(G\_\text{loss}\right). \end{array}$$

The discriminative training network is defined as

(13) $$\begin{array}{c} \text{Train}\_D=\text{optimizer}\left(\text{LR}\right).\text{minimize}\left(D\_\text{loss}\right). \end{array}$$

#### 4.2.3. Define Loss Function

The loss of the discriminative network needs to optimize the probability of the original line segment and the new line segment at the same time, so we get

(14) $$\begin{array}{c} D\_\text{loss}=-tf.\text{reduce}\_\text{mean}\left(tf.\;\log\left(\text{prob}\_\text{real}\right)+tf.\;\log\left(1-\text{prob}\_\text{new}\right)\right). \end{array}$$

By repeating the sentences of inputting new curves in the cyclic discriminant network, the loss of the discriminant network can be minimized by dynamically adjusting the weights. In the loss of the generation network, because there is no real curve input, only the probability value “prob_new” corresponding to the newly generated line segment needs to be used for calculation.

#### 4.2.4. Training and Model Saving

In the beginning of the loop, the newly generated packaging image will be significantly different from the original packaging image, which cannot fool the discriminant network, resulting in a large loss of function calculation. To prevent abnormal convergence of the generative network, the discriminative network learning rate needs to be set to 5–10 times the generative network learning rate. That is, after the discriminant network is trained for 5–10 times, the update training of the generation network will be performed once.

In terms of data protection, it is set to save a record point every 500 cycles, and a picture containing 64 icon samples is saved every 50 cycles. If the training process is stopped due to computer crash or insufficient memory, the saved record points can be reread for training.

In order to better observe the experimental results and the changes in loss function, the built-in tensorfboard visualization tool of tensorflow can be used. When using Tensorboard, we insert the “tf.summary” summary function into the relevant numerical definition program of the network model. After training, we will get the “logs” folder and the “evvents.out” file in the file directory. Right-click the terminal operation of the logs folder, write the program language for reading the log file, and wait for a moment to get the result immediately. Copy the IP address output from the terminal result to a local browser to open it and enter the visualization workbench. Copy the IP address output from the terminal result to a local browser to open it and enter the visualization workbench.

RETRACTED

As shown in Figure 4, in the Tensorboard interface, the left side is the display options of the line graph, including the setting of smoothness, relative interval, and boundary. The right side is the main display area, which supports general operations such as zooming, positioning, restoring, and downloading data.

#### 4.2.5. Training Results and Analysis

As shown in Figure 5, the loss of the discriminant network and the generation network will fluctuate drastically at several identical loop nodes. The loss peak of the discriminative network appears in the initial stage, which is 5.00, which is a high value, indicating that the discriminative network in the initial stage does not distinguish the real and newly generated packages very well. As the training loop increases, the loss of the discriminative network stabilizes around 0.20, and the average of the comprehensive loss is equal to 0.40.

Figure 6 shows the change in the loss of the generation network, which is in a fluctuating state most of the time, the loss value is up to 14.50, and the average error is 8.00.

As shown in Figure 7, after about 200 cycles, the output result gradually evolves from a bunch of noise points to a packaged image, with rich colors and mostly gradient mixed color blocks. The overall image performance is far from the actual icons, and it is impossible to distinguish the indications between different icons. Most of the packaging designs have the problem of collapsed and blurred graphics and do not show any clear instructions.

Using the DCGAN proposed in this paper to assist the appearance design of packaging products has a better effect, and the generated images are not only diverse but also have clear edges and rich colors; compared with the target image, the output image of the cloth tote bag has more colors and different patterns. The output image of the plastic environmental protection bag not only retains some details of the target image but also tries to give different color matching references on this basis; the output image of the paper portable gift box provides richer paper colors and the matching scheme of different patterns, and different color and pattern designs are given; the output image is richer in color, and the color matching is also very reasonable.

Finally, three schemes are screened out from the pictures generated by the DCGAN model generator and compared with the design schemes designed by three experts in two groups, as shown in Figure 8. It can be seen that when the number of iterations is 200, the satisfaction rates of the three schemes are 77%, 72%, and 67%, respectively, and the satisfaction rates of the three expert design schemes are 81%, 74%, and 71%, respectively. Among the three schemes, the design results based on DCGAN model are slightly less satisfactory than that of the expert design scheme.

RETRACTED

Tables 1 and 2 compare the peak signal-to-noise ratio (PSNR) and structural similarity index (SSIM) of the output image between the method proposed in this paper and the Pix2Pix algorithm. Higher PSNR and SSIM values indicate better quality of the output image.

It can be seen that the DCGAN method proposed in this paper achieves higher image output quality. It is feasible to apply this model to the appearance design of packaging products.

### 4.3. Experiment Results of Image Enhancement Effect in Packaging Design

In order to verify the enhancement ability of packaging design images of visual communication technology, experimental test analysis is carried out. It is assumed that the sampling sequence length of packaging design images under visual communication technology is 25, the number of training samples is 13, the grayscale feature decomposition coefficient is 0.35, and the window size is 12 × 24. According to the above parameter settings, the packaging design image enhancement processing under the visual communication technology is performed, and the image to be processed is obtained as shown in Figure 9.

Taking the packaging design image in Figure 8 as the test object, the information enhancement processing is carried out, the multidimensional scale feature decomposition of the packaging design image under the visual communication technology is carried out through the methods of visual communication optimization and edge pixel fusion, and the image filtering result is shown in Figure 9.

According to the filtering results in Figure 10, the packaging design image enhancement under the visual communication technology is carried out, and the enhancement results are shown in Figure 11. Figure 11 shows that the method in this paper can effectively realize the visual information enhancement processing of packaging design images under the visual communication technology and improve the visual expression ability of packaging images.

The output signal-to-noise ratio of the enhanced packaging design image under the visual communication technology is tested, and the comparison results are shown in Table 2. It can be seen from Table 2 that the output signal-to-noise ratio of the packaging design image enhancement processing under the visual communication technology by the method in this paper is high, indicating that the visual information enhancement ability is good.

RETRACTED

## 5. Conclusion

This paper proposes a packaging design model constructed using the DCGAN feature. By learning the packaging image data set, the DCGAN algorithm is used to quickly generate innovative packaging design schemes. Finally, in order to obtain the ideal packaging design image enhancement efficiency and improve the packaging design image quality, this paper uses the guided filtering method to enhance the packaging design image in the multiresolution visual imaging environment and establishes an optimized feature matching model for the packaging design image. The experimental results show that the model can effectively realize the innovative design of packaging, solve the problems of subjective tendencies and lack of overall consideration in traditional packaging design methods, and provide new ideas for the innovative design of packaging solutions. The output signal-to-noise ratio of the packaging design image enhancement processing method in this paper is high, and the obtained packaging image enhancement performance is better. The follow-up research mainly focuses on the following aspects: covering more types of packaging designs; further optimizing and improving the DCGAN design model.

## Figures and Tables

**Figure 1:** The structure of the generative adversarial network.

**Figure 2:** Packaging design dataset (part of example).

**Figure 3:** The basic framework of the packaging design generative adversarial network.

**Figure 4:** Tensorboard working interface.

**Figure 5:** Loss change of discriminant network.

**Figure 6:** Loss variation of the generative network.

**Figure 7:** Sample packaging images generated after 200 cycles. (a) 30th cycle. (b) 60th cycle. (c) 200th cycle.

**Figure 8:** Comparison of design satisfaction rates.

**Figure 9:** Image of packaging design to be processed.

**Figure 10:** Filtering results.

**Figure 11:** Image enhancement results.

**Table 1:** Comparison of PSNR values.

Algorithm	Output image sequence					Average value
	1	3	5	7	9	
DCGAN	13.7472	14.3874	16.3828	15.3843	17.3841	15.45
GAN	12.3841	14.2839	13.4858	14.8184	15.2335	14.04
Pix2Pix	10.3288	12.4821	10.3499	14.8310	13.8583	12.37

**Table 2:** Comparison of signal-to-noise ratios for image enhancement in packaging design (unit: dB).

Number of iterations	The method of this paper	Method of literature [10]	Method of literature [11]	Method of literature [12]
100	44.3	20.3	26.5	18.1
200	46.5	23.2	28.0	18.3
300	50.1	24.3	31.2	19.2
400	53.5	26.5	34.8	21.4

## Data Availability

The dataset can be accessed upon request.
